The article "The Disparity in the Management of Polycystic Ovary Syndrome between Obstetrician-Gynecologists in Different-Level Hospitals under the Hierarchical Medical System" was retracted in 2024. Reasons: signs of a paper mill; suspected computer-generated content; unreliable results or conclusions; concerns about the data.

# The Disparity in the Management of Polycystic Ovary Syndrome between Obstetrician-Gynecologists in Different-Level Hospitals under the Hierarchical Medical System

**DOI:** 10.1155/2022/9778678

**Published:** 2022-09-15

**Authors:** Yue Wang, Jie Chen, Han Dong, Ruilin Ma, Ying Zou, Wei Wang, Qingmei Zheng, Ying Feng, Zhangyun Tan, Xiaoqin Zeng, Yinqing Zhao, Yan Deng, Yanfang Wang, Bei Gu, Aijun Sun

**Affiliations:** ^1^Department of Obstetrics and Gynecology, Peking Union Medical College Hospital, Chinese Academy of Medical Sciences and Peking Union Medical College, Beijing 100730, China; ^2^Department of Obstetrics and Gynecology, Women and Children's Hospital of Jinzhou, Jinzhou, 121000 Liaoning, China; ^3^Department of Obstetrics and Gynecology, Hunan Provincial Maternal and Child Health Care Hospital, Changsha, 410008 Hunan, China; ^4^Department of Reproductive Medicine, The Second Hospital of Hebei Medical University, Shijiazhuang, 050000 Hebei, China; ^5^Department of Gynecology, The Affiliated Hospital of Qingdao University, Qingdao, 266500 Shandong, China; ^6^Department of Obstetrics and Gynecology, The Second Affiliated Hospital of Nanchang University, Nanchang, 330006 Jiangxi, China; ^7^Department of Obstetrics and Gynecology, Xinhui Maternity and Children's Hospital, Nanning, 529100 Guangxi, China; ^8^Department of Gynecology, Guangzhou Women and Children's Medical Center, Guangzhou, 510000 Guangdong, China; ^9^Department of Obstetrics and Gynecology, Beijing Shijitan Hospital, Capital Medical University, Peking University Ninth School of Clinical Medicine, Beijing 100038, China; ^10^Department of Obstetrics and Gynecology, Peking Union Medical College Hospital, Beijing 100010, China

## Abstract

**Background:**

PCOS is a prevalent endocrine and metabolic disorder in women characterized by abnormal blood glucose, dyslipidemia, and abnormal mental health. To improve patient care, the goal of our study is to find out if there are differences in how PCOS patients are treated at different hospital levels within the hierarchical medical system.

**Methods:**

Obstetricians and gynecologists from primary, secondary, and tertiary hospitals were the participants in the survey. The responses provided and collected were analyzed using various statistical techniques like the chi-square test, Fisher exact test, and logistic regression with multiple variables.

**Results:**

The investigation examined 2298 survey replies (13.1% primary hospitals, 52.4% secondary hospitals, and 34.5% tertiary hospitals). As hospital grade increases, more participants inquire about a patient's history of unfavorable pregnancies concerning hormone evaluation; the better the hospital's grade, the greater the number of participants who would undergo AMH and androgen-related tests. The higher the hospital level, the more participants would pick the oral glucose tolerance test (OGTT) to determine insulin resistance, the BMI Asian criteria for defining obesity, and blood lipids. Participants in primary (odds ratio (OR) = 0.383, 95% confidence interval (CI) 0.282-0.520) and secondary (OR = 0.607, 95% confidence interval (CI) 0.481-0.765) hospitals were significantly less likely to select OGTT than those in tertiary hospitals. Comparatively, fewer primary hospitals chose to do lipid profiling than tertiary hospitals (OR 0.689, 95% CI 0.523-0.909). With the increase in hospital level, participants were more knowledgeable about the multiple efficacies and dose alternatives of metformin and selected letrozole and assisted reproduction more frequently.

The article "The Disparity in the Management of Polycystic Ovary Syndrome between Obstetrician-Gynecologists in Different-Level Hospitals under the Hierarchical Medical System" was retracted in 2024. Reasons: signs of a paper mill; suspected computer-generated content; unreliable results or conclusions; concerns about the data.

**Conclusion:**

Our study uncovered differences in the endocrine evaluation, metabolic screening, and management of PCOS patients across obstetrics and gynecology at various hospital levels. Simultaneously, it underlines the need to improve the hierarchical medical system and close the knowledge gap across hospitals.

## 1. Introduction

Polycystic ovary syndrome (PCOS) is one of the women's most prevalent reproductive endocrine diseases, affecting 9-18% of females [1–3]. Clinically, women with PCOS are widely dispersed across age groups, exhibiting diverse symptoms and prominent genetic traits. Patients with different needs necessitate individualized treatment strategies, posing new difficulties in diagnosing and treating the disease.

PCOS's pathogenesis is complex. Genetic and environmental factors alter the signaling pathway of the hypothalamic-pituitary-ovarian axis, thereby promoting ovarian and adrenal hyperandrogenism. Insulin resistance (IR), adipose tissue accumulation, and lipid toxicity exacerbate PCOS. The dysfunction of oxidative stress also worsens symptoms [4]. Independent of BMI, women with PCOS have a threefold higher risk of impaired glucose tolerance [5], particularly in Asia and North and South America. There is a strong relationship between obesity and PCOS prevalence [6]. According to a large-scale, high-quality meta-analysis, the risk of obesity in women with PCOS is four times that of women without the condition. White women are more likely to be obese than Asian women [7]. According to Dumesic et al., the prevalence of PCOS increased significantly among women with a BMI greater than 30 kg/m^2^ [4]. Hyperandrogenism and obesity have been linked to several psychological disorders [8, 9]. In cross-sectional studies, moderate to severe depression and anxiety symptoms have increased [10]. Several longitudinal studies, meanwhile, have reached similar conclusions [11]. Thus, the syndrome encompasses metabolic, reproductive, and psychological disorders.

The article "The Disparity in the Management of Polycystic Ovary Syndrome between Obstetrician-Gynecologists in Different-Level Hospitals under the Hierarchical Medical System" was retracted in 2024. Reasons: signs of a paper mill; suspected computer-generated content; unreliable results or conclusions; concerns about the data.

PCOS is identified based on three specific factors: oligoovulation, clinical or biochemical androgen excess, and ultrasound assessment of ovarian morphology. Currently, there is no definitive diagnostic model for PCOS. The evidence-based international guidelines [12] endorse the Rotterdam criteria as an exclude-diagnosis. The requirements suggest excluding thyroid diseases, hyperprolactinemia, and atypical congenital adrenal hyperplasia (screening with 17-hydroxyprogesterone) and meeting two of the three diagnostic criteria [13] for the diagnosis of adult women. In Asian women, hyperandrogenism manifests primarily as skin manifestations, such as hirsutism (modified Ferriman-Gallwey (mFG) score), acne, and alopecia [14]. Neither biologically nor clinically is pelvic ultrasound required to diagnose women with menstrual irregularities and hyperandrogenism. The clinical diagnosis is still valid even without a comprehensive ultrasound morphological evaluation. Levels of AMH have been considered as an alternative biomarker for diagnosing polycystic ovary morphology (PCOM), or ultrasound follicle number per ovary (FNPO) counts, as well as an independent marker for PCOS [15]. The total serum AMH level in women with PCOS is two to three times that of women with normal reproductive function, and this level correlates with FNPO ultrasound measurements. Several studies have demonstrated that the median level of AMH in PCOS women is 20-81.6 pmol/L, whereas it ranges from 16.7 to 33.5 pmol/L in normal controls [16, 17]. Lifestyle modification is the most fundamental treatment that can somewhat alleviate symptoms [18–20]. Oral contraceptives, metformin, and GLP-1 receptor agonist have demonstrated respective advantages in drug therapy [21–23].

The hierarchical medical system classifies hospitals into three levels based on size, scientific research direction, skills, technical prowess, and medical equipment. Several studies [24] demonstrate that primary (community) hospitals play indispensable roles in the early diagnosis, treatment, and long-term management of common diseases such as PCOS. Consequently, the only way to improve diagnosis and treatment technology is to acknowledge the disparity between hospitals of all grades. To promote evidence-based medicine and standardize the diagnosis, treatment, and management of PCOS women, our study seeks to identify disparities in hospital management from various perspectives.

## 2. Methods

### 2.1. Study Design, Setting, and Participants

A countrywide online survey was performed between 1 and 30 September 2020. Physicians who had joined the China Maternal and Child Health Association's online chat groups received an invitation to accept and complete an online questionnaire intended for this purpose, along with instructions and a web link. All individuals were encouraged to participate voluntarily while maintaining their anonymity. Participants' consent to participate in the study was assumed when they completed the survey.

The article "The Disparity in the Management of Polycystic Ovary Syndrome between Obstetrician-Gynecologists in Different-Level Hospitals under the Hierarchical Medical System" was retracted in 2024. Reasons: signs of a paper mill; suspected computer-generated content; unreliable results or conclusions; concerns about the data.

### 2.2. Questionnaire Content

The questionnaires inquired about the demographics, clinical specialties, hospital levels, practice attributes, obesity and IR diagnostic criteria, provider knowledge of obesity, and PCOS evaluation and treatment, as well as weight reduction and treatment procedures for women with PCOS. The questionnaire was piloted with thirty obstetricians and gynecologists, and their feedback was considered; its content was clear and concise.

### 2.3. Ethical Approval

Prior to initiation, the study protocol was approved by the Ethics Committee of Peking Union Medical College Hospital, Chinese Academy of Medical Sciences, China, per protocol number S-K1373.

## 3. Statistical Analysis

SPSS was used to evaluate the collected data (version 23.0, IBM, Armonk, NY, USA). Frequencies and percentages were used to present categorical data. We used the procedures of Ma et al. [25], comparing various groups using Pearson's *χ*^2^ tests or Fisher's exact tests, depending on the situation. In a multivariable logistic regression analysis, physician gender, specialty, age, hospital grade, the number of PCOS patients seen annually, and the proportion of PCOS women with obesity and insulin resistance (IR) were considered. Statistical significance was defined as a *p* value of less than 0.05.

## 4. Results

A total of 2509 questionnaires were completed and submitted by the participants. Among these, 211 questionnaires completed by nonobstetricians and gynecologists were excluded, resulting in the remaining 2298 questionnaires in the final analysis.

### 4.1. General Characteristics of the Participants

The general information of patients is shown in Table 1, of which 13.1% are from primary hospitals, 52.4% from secondary hospitals, and 34.5% from tertiary hospitals. Among the participants in the survey, 98.2% (2,256) were female, and 1.8% (42) were male. The proportion of male doctors increased as the grade of hospitals increased. More than 80% of participants were over 35 years old, while a total of 181 (7.9%) were reproductive endocrinologists (Repro-Endo), and 2,117 (92.1%) were nonreproductive endocrinologists in obstetrics and gynecology (Ob-Gyn). The proportion of reproductive endocrinologists in tertiary hospitals increased significantly (15.5%). In tertiary hospitals, the majority of participants admitted 0-50 PCOS patients annually, but over 40% of participants saw more than 50 patients annually. The chief paramount complaints of patients were menstrual disorder (79.8%) and infertility (17.6%). Moreover, a small number of patients were also treated for acne, acanthosis nigricans, abnormal blood glucose, obesity, and other reasons. Regarding understanding PCOS complications, most participants (60.8%) thought about 0-30% of PCOS patients combined with IR. With the grade of the hospital increase, doctors reckoned the proportion of patients combined with IR would be higher (*p* < 0.001), and about half (47.4%) of tertiary hospital doctors believe IR prevalence > 30%. Most doctors (72.1%) thought that the probability of PCOS combined with obesity was 0-50%. With the improvement of hospital grades, doctors generally believed that the prevalence of PCOS combined with obesity increased (*p* < 0.001).

The article "The Disparity in the Management of Polycystic Ovary Syndrome between Obstetrician-Gynecologists in Different-Level Hospitals under the Hierarchical Medical System" was retracted in 2024. Reasons: signs of a paper mill; suspected computer-generated content; unreliable results or conclusions; concerns about the data.

### 4.2. Diagnosis and Evaluation of PCOS Patients

The international evidence-based guidelines [13] endorse using the Rotterdam criteria for diagnosing PCOS, but a comprehensive evaluation is necessary for newly diagnosed patients, a thorough review, including the history of hormone and metabolic assessment. In the aspect of medical history inquiry (Table 2), different doctors may emphasize PCOS as it is affected by many factors. Almost all participants noticed whether patients had a family history of diabetes (95.2%) and PCOS (88.6%), and 82.7% of participants asked patients whether they had a history of adverse pregnancy and delivery, which was particularly prominent in tertiary hospitals (*p* = 0.041). Most participants also noted a history of thyroid diseases (77.9%), cardiovascular disease, and family history (66.1%). 53.5% of participants would pay attention to patients' mental health, asking whether they have anxiety or depression, and there is no significant statistical difference between different grades of hospitals. Almost all participants (98.7%) underwent six sex hormone tests (Figure 1).

In addition, AMH (57.8%) and other androgen-related indicators such as androstenedione, dehydroepiandrosterone sulfate, and free testosterone (57.2%) were also assessed by some physicians. With the increase in hospital grade, more participants set these hormone levels (*p* < 0.001). The most common metabolic abnormalities associated with PCOS are IR, obesity, and dyslipidemia. The evaluation of metabolic abnormalities is shown in Table 2 and Figure 2. The gold standard for IR diagnosis is the OGTT test. About half of the participants (48.8%) most often chose OGTT for IR diagnosis, and the number of participants increased successively from the primary, secondary, and tertiary hospitals (*p* < 0.001). In addition, some participants also chose to fast blood glucose and blood insulin (21.9%), 2 hours postprandial blood glucose and blood insulin (12.9%), and HOMA-IR (5.6%) for diagnosis. The evaluation criteria for obesity mainly included BMI and waist circumference. Most participants would choose the BMI China standard (59%) for evaluation, but participants in tertiary hospitals (14.1%) would also adopt BMI Asian standard (*p* = 0.001). Only a minority (1.3%) of participants would choose waist circumference > 80 cm to assess obesity, and there was no significant difference between hospitals.

The article "The Disparity in the Management of Polycystic Ovary Syndrome between Obstetrician-Gynecologists in Different-Level Hospitals under the Hierarchical Medical System" was retracted in 2024. Reasons: signs of a paper mill; suspected computer-generated content; unreliable results or conclusions; concerns about the data.

In univariate analysis, physicians who specialized in reproductive endocrinology had an estimated prevalence of overweight/obesity at 31-80%, and an estimated prevalence of IR >30% was more likely to perform OGTT on PCOS patients. Physicians who specialized in reproductive endocrinology and estimated an IR prevalence of greater than 30 percent were more likely to order lipid profiling for PCOS patients. Participants in primary (odds ratio (OR) 0.383, 95% confidence interval (CI) 0.282-0.520) and secondary (OR 0.607, 95% confidence interval (CI) 0.481-0.764) hospitals were less likely to select OGTT than those in tertiary hospitals. Compared with the tertiary hospital group, fewer primary hospitals chose to perform lipid profiling (OR 0.689, 95% CI 0.523-0.909) (Table 3).

### 4.3. Treatment and Management of PCOS

PCOS treatment has different needs for women of different ages (Figure 3). Most participants recognize that lifestyle intervention and weight management are the most basic treatment options. Regarding drug therapy, most participants believed that metformin could be used regardless of the patient's need for fertility.  Figure 4 shows the dose selection of metformin. With the increase in hospital grade, physicians would be more active in their choice, preferring 1 g/day or 1.5 g/day. About 1/10 of participants were unclear about the dose selection of metformin, as was 1/5 (22.9%) in the primary hospital group. Most participants (63.8%) of patients without fertility needs believed that oral contraceptives could be used for a long time by regularly checking liver and kidney functions. There was no significant difference among different level hospitals. Some participants agreed to use letrozole, assisted reproductive technology (ART), for patients with fertility needs. The higher the hospital level, the higher the proportion of participants who chose this program. In terms of weight loss, in addition to dietary adjustment, metformin and orlistat were preferred by more physicians with the increase in hospital grade. Some participants in primary hospitals tried traditional Chinese medicine weight loss programs (Figure 5). PCOS is a metabolic disease caused by endocrine disorders under multiple factors, which requires the cooperation and long-term management of hospitals and patients. However, participants also generally reported that patients did not understand the disease well in receiving treatment.

The article "The Disparity in the Management of Polycystic Ovary Syndrome between Obstetrician-Gynecologists in Different-Level Hospitals under the Hierarchical Medical System" was retracted in 2024. Reasons: signs of a paper mill; suspected computer-generated content; unreliable results or conclusions; concerns about the data.

## 5. Discussion

The hierarchical medical system contributes to the hierarchical management of diseases and resolves the problem of individuals' difficulty in obtaining medical care. Simultaneously, hospitals at all levels carry out their respective responsibilities, thereby enhancing the efficacy of disease diagnosis and treatment, conserving medical resources to some extent, and maximizing the utilization rate of medical resources. Nonetheless, the hierarchical medical system inevitably produces disparities in hospital diagnosis and treatment, particularly for chronic diseases with multiple manifestations and complications, such as PCOS. A lack of reproductive endocrinology specialists, coupled with the fact that primary hospitals treat far fewer patients annually than tertiary hospitals, has led to the current situation in which primary hospital group participants have a limited understanding of diseases. Regarding physician composition, secondary hospitals have the most significant number of participants, which meets the requirements of China's current diagnosis and treatment model. The majority of participants in primary hospitals are female. As hospital conditions improve, the proportion of male obstetricians and gynecologists gradually increases. In terms of age composition, the majority of primary hospital physicians are older. This phenomenon demonstrates that tertiary hospital physicians have shattered the stereotype that “obstetricians and gynecologists are all female physicians” and that an increase in the number of young physicians indicates a greater willingness to update knowledge and engage in lifelong learning. As the hospital level increased, participants generally agreed that PCOS patients had a higher incidence of insulin resistance and obesity, which was helpful in alerting physicians to this aspect of patient assessment. This serves as a reminder to primary care physicians to pay attention to the advancement of research and the updating of their knowledge; tertiary hospitals should also assist primary hospitals in times of difficulty and establish an effective chronic disease cooperative management mechanism.

The article "The Disparity in the Management of Polycystic Ovary Syndrome between Obstetrician-Gynecologists in Different-Level Hospitals under the Hierarchical Medical System" was retracted in 2024. Reasons: signs of a paper mill; suspected computer-generated content; unreliable results or conclusions; concerns about the data.

Almost all participants were concerned about whether or not patients had a family history of diabetes, PCOS, and thyroid-related diseases. However, less than two-thirds of the participants paid attention to a cardiovascular disease history. Insulin resistance is typically involved in the pathogenesis of polycystic ovary syndrome (PCOS), leading to various cardiometabolic abnormalities (such as dyslipidemia, hypertension, glucose intolerance, diabetes, and metabolic syndrome) and thereby increasing the risk of cardiovascular disease in women [26]. Most doctors also inquired about a patient's history of adverse pregnancies, and as hospital grades improved, more participants inquired. The study by Palomba et al. demonstrated that PCOS patients are more likely to experience pregnancy complications, which endanger the mother's and fetus's health. Only fifty percent of participants would inquire about the patients' mental health. Current research indicates that dysfunction of the H-P-O axis may involve a broader range of functional brain regions and lead to psychological and emotional issues [8, 9].

In assessing patients' specific conditions, hospitals of varying acuity also have unique characteristics. Regarding the selection of obesity standards, most physicians use the BMI China standard to define obesity. Some participants in tertiary hospitals will also choose the stricter BMI Asian standard for definition, which can identify high-risk obese individuals earlier than the BMI China standard. Few participants selected a waist circumference greater than 80 cm as the standard for obesity. The waist circumference can effectively detect abdominal obesity in patients, and abdominal obesity in PCOS patients frequently indicates a greater metabolic risk. However, abdominal obesity is not an absolute measure of obesity; instead, it serves as a supporting factor. At this time, there is no evidence indicating which obesity criteria are more effective at predicting the comorbidities of PCOS patients, and more research is required in this area. OGTT is the gold standard for evaluating blood glucose and measuring blood glucose.

Nonetheless, in actual clinical practice, the higher the hospital level, the greater the number of participants who choose OGTT, and the choice of OGTT is also dependent on the time and patient compliance during the administration of this examination. Less than one-third of the participants assessed all patients for IR. Existing studies indicate that IR is independent of obesity, and patients are at particular risk of IR regardless of whether they are overweight or lean [27, 28]. In addition, physicians in tertiary hospitals are more willing to experiment with new blood glucose assessment techniques, such as HOMA-IR. Regarding the assessment of sex hormones, nearly all participants in hospitals at all levels would conduct a six-item evaluation of sex hormones. In addition, more physicians at tertiary hospitals evaluate AMH and other androgens, including androstenedione, dehydroepiandrosterone sulfate, and free testosterone. According to studies, AMH plays an essential role in the early detection of PCOS, and it is independent of BMI and resistant to interference from other factors. The increase of androstenedione (AED), dehydroepiandrosterone sulfate (DHEAS), and free testosterone (T), particularly DHEAS, was observed as a result of abnormalities of androgen precursors in the general population and women with PCOS, according to studies [29]. Increased androgen levels may play a role in preventing cardiovascular disease, but there are currently no conclusive studies on this topic. Several metabolic abnormalities characterize PCOS, and patients with additional needs may require specialized examinations. A comprehensive assessment of the patient's condition is essential for newly diagnosed patients.

The article "The Disparity in the Management of Polycystic Ovary Syndrome between Obstetrician-Gynecologists in Different-Level Hospitals under the Hierarchical Medical System" was retracted in 2024. Reasons: signs of a paper mill; suspected computer-generated content; unreliable results or conclusions; concerns about the data.

Participants in all hospitals were aware that lifestyle modification and weight loss are the most effective treatment strategies. Most participants agreed that timely treatment of PCOS patients with metformin and GLP-1 agonists would help alleviate symptoms. Studies have demonstrated that the benefits of GLP-1 receptor agonists are not limited to the improvement of insulin sensitivity (IR) but also include weight loss and androgen reduction [30]. Although most participants chose metformin, hospital doses varied considerably. Community hospitals were more likely to use a dose of 0.5 g/day, whereas higher-level hospitals were more likely to use a dose of 1.0-1.5 g/day. According to the American Society of Clinical Endocrinology [31], metformin is the first-line treatment for PCOS, with a recommended dosage of 0.85 g/day for patients of normal weight and 1.5-2.5 g/day for those with a higher BMI. Various treatments also depend on whether or not the patient desires to reproduce. After diagnosing infertility, most participants chose oral contraceptives for patients without reproductive needs; if patients have fertility needs, the majority of participants recommended assisted reproductive technology. Additional large-scale clinical trials of alternative treatments and drug combinations are required to improve comorbidities [32, 33].

## 6. Conclusions

This was the most comprehensive survey of PCOS disease management in hospitals of varying grades under the hierarchical medical system. This survey reflects the characteristics and benefits of a hierarchical medical system by comparing the differences in diagnosing and treating PCOS diseases at various hospital levels. This facilitates identifying potential issues and improving diagnosis and treatment standards within China's tertiary hospital system. Despite this, the survey has limitations. First, participants were distributed unevenly by gender and hospital grade. Second, the age of PCOS patients with IR or obesity was not recorded. Lastly, we did not track specific drug combinations. Consequently, additional research is required to confirm and update our conclusions.

The article "The Disparity in the Management of Polycystic Ovary Syndrome between Obstetrician-Gynecologists in Different-Level Hospitals under the Hierarchical Medical System" was retracted in 2024. Reasons: signs of a paper mill; suspected computer-generated content; unreliable results or conclusions; concerns about the data.

Our findings revealed disparities in the knowledge of metabolic screening for PCOS patients at various hospital levels and differences in assessing and treating participants. Tertiary hospitals have a complete set of diagnosis and treatment standards, so the evaluation is adequate. In contrast, primary hospitals are more open to integrating traditional Chinese and western medicine treatment methods, such as traditional Chinese medicine for weight loss. Secondary hospitals fall between the primary and tertiary hospitals. It also emphasizes the significance of early standardization and comprehensive evaluation of PCOS patients. To narrow the differences in the management of PCOS disease, it is recommended that tertiary hospitals conduct more communication activities in the form of knowledge lectures. Simultaneously, all participants should update their self-knowledge, actively monitor research progress, and improve patient care.

## Figures and Tables

**Figure 1:** Hormonal level estimation for PCOS patients in different grades of hospitals. SH: sex hormone test (including FSH, LH, estradiol, testosterone, PRL, and progestin); AMH: anti-Müllerian hormone; AH: androgenic hormone test (including androstenedione, dehydroepiandrosterone sulfate, and free testosterone). Primary vs. secondary hospital (^✭^*p* < 0.05 and ^✭✭^*p* < 0.001). Primary vs. tertiary hospital (^✸^*p* < 0.05 and ^✸✸^*p* < 0.001). Secondary vs. tertiary hospital (^◆^*p* < 0.05 and ^◆◆^*p* < 0.05).

**Figure 2:** Patients with PCOS results of OGTT, FPG, and FINS. Primary vs. secondary hospital (^✭^*p* < 0.05). Primary vs. tertiary hospital (^✸^*p* < 0.05 and ^✸✸^*p* < 0.001). Secondary vs. tertiary hospital (^◆^*p* < 0.05 and ^◆◆^*p* < 0.05). OGTT = oral glucose tolerance test; FPG = fasting plasma glucose; FIN = fasting insulin.

**Figure 3:** Treatment recommendations for women with PCOS. Primary hospital vs. secondary hospital (^✭^*p* < 0.05 and ^✭✭^*p* < 0.001). Primary hospital vs. tertiary hospital (^✸^*p* < 0.05 and ^✸✸^*p* < 0.001). Secondary hospital vs. tertiary hospital (^◆^*p* < 0.05 and ^◆◆^*p* < 0.05).

The article "The Disparity in the Management of Polycystic Ovary Syndrome between Obstetrician-Gynecologists in Different-Level Hospitals under the Hierarchical Medical System" was retracted in 2024. Reasons: signs of a paper mill; suspected computer-generated content; unreliable results or conclusions; concerns about the data.

**Figure 4:** Most common dosage of metformin prescribed in women with PCOS.

**Figure 5:** The recommended method of weight loss for women with PCOS. GLP-1 receptor agonist, glucagon-like peptide-1 receptor agonist.

**Table 1:** General information provided by the study participants.

	Overall (*n* = 2298)	Primary hospital (*n* = 301)	Secondary hospital (*n* = 1204)	Tertiary hospital (*n* = 793)	*p* value
Sex					
Female	2256 (98.2)	300 (99.7)	1192 (99.0)	764 (96.3)	<0.001
Male	42 (1.8)	1 (0.3)	12 (1.0)	29 (3.7)	<0.001
Age					
18-35	335 (14.6)	28 (9.3)	120 (10.0)	187 (23.6)	<0.001
36-45	890 (38.7)	124 (41.2)	466 (38.7)	300 (37.8)	NS
>45	1073 (46.7)	149 (49.5)	618 (51.3)	306 (38.6)	<0.001
Specialty					
Ob-Gyn	2117 (92.1)	296 (98.3)	1151 (95.6)	670 (84.5)	<0.001
Repro-Endo	181 (7.9)	5 (1.7)	53 (4.4)	123 (15.5)	<0.001
No. of patients with PCOS treated annually					
<50	1649 (71.8)	269 (89.4)	915 (76.0)	465 (58.6)	<0.001
50-200	511 (22.2)	24 (8.0)	247 (20.5)	240 (30.3)	<0.001
>200	138 (6.0)	8 (2.6)	42 (3.5)	88 (11.1)	<0.001
The chief complaint about clinic attendance in patients with PCOS					
Menstrual disorders	1833 (78.9)	223 (74.1)	957 (79.5)	653 (82.3)	0.009
Infertility	405 (17.6)	67 (22.2)	217 (18.0)	121 (15.4)	<0.001
Obesity/IR	39 (1.7)	5 (1.7)	17 (1.4)	17 (2.1)	0.017
Hirsutism/acne	14 (0.6)	5 (1.7)	8 (0.7)	1 (0.1)	0.013
Others	7 (0.3)	1 (0.3)	5 (0.4)	1 (0.1)	NS
Estimated national prevalence of IR in patients with PCOS (%)					
0-30	1398 (80.8)	211 (70.1)	766 (63.8)	419 (52.8)	<0.001
31-60	754 (32.8)	72 (23.9)	382 (31.8)	300 (37.8)	<0.001
>60	146 (6.4)	18 (6.0)	54 (4.4)	74 (9.4)	<0.001
Estimated national prevalence of obesity in patients with PCOS (%)					
0-30	748 (32.6)	142 (47.2)	387 (32.1)	219 (27.6)	<0.001
30-50	909 (39.5)	87 (26.9)	495 (41.1)	327 (41.2)	<0.001
50-80	522 (22.7)	51 (16.9)	254 (21.2)	217 (27.4)	<0.001
>80	119 (5.2)	21 (7.0)	68 (5.6)	30 (3.8)	NS

Ob-Gyn = obstetrician-gynecologists (specialization outside of reproductive medicine); Repro-Endo = reproductive endocrinologists; PCOS = polycystic ovary syndrome; IR = insulin resistance; NS = not significant.

**Table 2:** Physicians' approach to patients' management suffering from obesity and PCOS.

	Overall (*n* = 2298)	Primary hospital (*n* = 301)	Secondary hospital (*n* = 1204)	Tertiary hospital (*n* = 793)	*p* value
Commonly used diagnostic criterion for IR.					
OGTT-insulin release test	1122 (48.8)	109 (36.2)	570 (47.3)	443 (55.9)	<0.001
Fasting insulin and blood glucose	503 (21.9)	74 (24.6)	280 (23.3)	149 (18.8)	0.029
Fasting and 2 h insulin and blood glucose	285 (12.4)	42 (14.0)	146 (12.1)	97 (12.2)	NS
HOMA-IR	128 (5.6)	15 (5.0)	64 (5.3)	49 (6.2)	NS
Other	260 (11.3)	61 (20.2)	144 (12.0)	55 (6.9)	<0.001
The diagnostic criterion used for obesity					
BMI (WHO criteria)	659 (28.7)	90 (29.9)	347 (28.8)	222 (28.0)	NS
BMI (Chinese criteria)	1355 (59.0)	187 (62.1)	719 (59.7)	449 (56.6)	NS
BMI (Asian criteria)	250 (10.9)	23 (7.6)	115 (9.6)	112 (14.1)	0.001
Measure waistline	31 (1.3)	1 (0.4)	21 (1.7)	9 (1.2)	NS
Other	3 (0.1)	0 (0)	2 (0.2)	1 (0.1)	NS
Family history of diabetes inquiry					
Yes	2188 (95.2)	284 (94.4)	1144 (95.0)	760 (95.8)	NS
Family history of PCOS inquiry					
Yes	2036 (88.6)	261 (86.7)	1069 (88.8)	709 (89.0)	NS
Family history of cardiovascular disease inquiry					
Yes	1518 (66.1)	189 (62.7)	793 (65.9)	536 (67.6)	NS
Family history of unfavorable pregnancy inquiry					
Yes	1889 (82.2)	233 (77.4)	993 (82.5)	663 (83.6)	0.041
Symptoms of anxiety, depression, and other psychological problems inquiry					
Yes	1229 (53.5)	166 (55.1)	630 (52.3)	433 (54.6)	NS

Abbreviations: IR = insulin resistance; OGTT = oral glucose tolerance test; HOMA-IR = homeostasis model assessment-insulin resistance; WHO = World Health Organization; PCOS = polycystic ovary syndrome; BMI = body mass index; NS = not significant.

The article "The Disparity in the Management of Polycystic Ovary Syndrome between Obstetrician-Gynecologists in Different-Level Hospitals under the Hierarchical Medical System" was retracted in 2024. Reasons: signs of a paper mill; suspected computer-generated content; unreliable results or conclusions; concerns about the data.

**Table 3:** Multinominal logistic regression analysis results of physician characteristics, OGTT, and lipid profile analysis for PCOS patients.

Variables	Physicians ordering OGTT	Physicians not ordering OGTT	Exp (B)	95% CI	Physicians ordering lipid profiles	Physicians not ordering lipid profiles	Ex (B)	95% CI
Sex								
Female	1750 (98.1)	506 (98.2)	0.943	(0.448, 1.984)	1503 (98.4)	753 (97.8)	1.357	(0.728, 2.529)
Male	33 (1.9)	9 (1.8)	1	1	25 (1.6)	17 (2.2)	1	1
Age								
18-35	273 (15.3)	62 (12.0)	1.437	(1.055, 1.957)^a^	204 (13.4)	131 (17.0)	0.767	(0.595, 0.988)^a^
35-45	701 (39.3)	189 (36.7)	1.210	(0.979, 1.497)^a^	605 (39.6)	285 (37.0)	1.047	0.866, 1.266)
≥46	809 (45.4)	264 (51.3)	1	1	719 (47.0)	354 (46.0)	1	1
Hospital grade								
1	201 (11.3)	100 (19.4)	0.383	(0.282, 0.520)^aa^	796 (52.1)	408 (53.0)	0.715	(0.715, 1.105)
2	916 (51.3)	288 (55.9)	0.607	(0.481, 0.764)^aa^	796 (52.1)	408 (53.0)	0.715	(0.715, 1.051)
3	666 (37.4)	127 (24.7)	1	1	549 (35.9)	244 (31.7)	1	1
Specialty								
Repro-Endo	152 (8.5)	29 (5.6)	1.562	(1.037, 2.353)^a^	142 (9.3)	39 (5.1)	1.920	(1.322, 2.768)^aa^
Ob-Gyn	1631 (91.5)	488 (94.4)	1		1386 (90.7)	731 (94.9)	1	1
Annual patients with PCOS								
<50	1240 (69.5)	409 (79.4)	0.638	(0.405, 1.005)	1083 (70.9)	566 (73.5)	0.837	(0.574, 1.220)
5-200	429 (24.1)	82 (15.9)	1.101	(0.668, 1.815)	349 (22.8)	162 (21.0)	0.943	(0.624, 1.417)
>200	114 (6.4)	24 (4.7)	1	1	96 (6.3)	42 (5.5)	1	1
The proportion of obesity in PCOS (%)								
0-30	535 (30.0)	213 (41.4)	1.047	(0.684, 1.601)	477 (31.2)	271 (35.2)	0.704	(0.460, 1.077)
31-50	743 (41.7)	166 (32.2)	1.865	(1.215, 2.863)^a^	609 (39.9)	300 (39.0)	0.812	(0.533, 1.237)
51-80	421 (23.6)	101 (19.6)	1.737	(1.107, 2.724)^a^	357 (23.4)	165 (21.4)	0.865	(0.558, 1.342)
>80	84 (4.7)	35 (6.8)	1	1	85 (5.5)	34 (4.4)	1	1
The proportion of IR in PCOS (%)								
0-30	1031 (71.3)	367 (71.3)	0.346	(0.203, 0.589)^aa^	903 (59.1)	485 (64.3)	0.642	(0.437, 0.944)^a^
30-60	622 (34.9)	132 (25.6)	0.580	(0.334, 1.007)	517 (33.8)	237 (30.8)	0.766	(0.514, 1.145)
>60	130 (7.3)	16 (3.1)	1	1	108 (7.1)	38 (4.9)	1	1

Abbreviations: Repro-Endo = reproductive endocrinologists; Ob-Gyn = obstetrician-gynecologists; PCOS = polycystic ovary syndrome; IR = insulin resistance. ^a^*p* < 0.05 and ^aa^*p* < 0.001.

The article "The Disparity in the Management of Polycystic Ovary Syndrome between Obstetrician-Gynecologists in Different-Level Hospitals under the Hierarchical Medical System" was retracted in 2024. Reasons: signs of a paper mill; suspected computer-generated content; unreliable results or conclusions; concerns about the data.

## Data Availability

The datasets used and/or analyzed during the current study are available from the corresponding author on reasonable request.
